This article has been retracted.

# MicroRNA-346-5p Regulates Differentiation of Bone Marrow-Derived Mesenchymal Stem Cells by Inhibiting Transmembrane Protein 9

**DOI:** 10.1155/2020/8822232

**Published:** 2020-11-22

**Authors:** Yicai Zhang, Yi Sun, Jinlong Liu, Yu Han, Jinglong Yan

**Affiliations:** ^1^Department of Orthopedic, The Second Affiliated Hospital of Harbin Medical University, Harbin, Heilongjiang, 150010, China; ^2^Department of Orthopedic, The Third People's Hospital of Huizhou, Huizhou, Guangdong, 516002, China; ^3^Department of Orthopedic, The 80th Group Army Hospital of PLA, Weifang, Shandong 261042, China

## Abstract

The molecular mechanisms how bone marrow-derived mesenchymal stem cells (BMSCs) differentiate into osteoblast need to be investigated. MicroRNAs (miRNAs) contribute to the osteogenic differentiation of BMSCs. However, the effect of miR-346-5p on osteogenic differentiation of BMSCs is not clear. This study is aimed at elucidating the underlying mechanism by which miR-346-5p regulates osteogenic differentiation of human BMSCs. Results of alkaline phosphatase (ALP) and Alizarin Red S (ARS) staining indicated that upregulation of miR-346-5p suppressed osteogenic differentiation of BMSCs, whereas downregulation of miR-346-5p enhanced this process. The protein levels of the osteoblastic markers Osterix and Runt-related transcription factor 2 (Runx2) were decreased in cells treated with miR-346-5p mimic at day 7 and day 14 after being differentiated. By contrast, downregulation of miR-346-5p elevated the protein levels of Osterix and Runx2. Moreover, a dual-luciferase reporter assay revealed that Transmembrane Protein 9 (TMEM9) was a target of miR-346-5p. In addition, the Western Blot results demonstrated that the TMEM9 protein level was significantly reduced by the miR-346-5p mimic whereas downregulation of miR-346-5p improved the protein level of TMEM9. These results together demonstrated that miR-346-5p served a key role in BMSC osteogenic differentiation of through targeting TMEM9, which may provide a novel target for clinical treatments of bone injury.

## 1. Introduction

It has been reported that BMSCs have potential for differentiation into the bone, cartilage, adipose tissue, and muscle [1]. Osteoporosis is a systemic skeletal disease with characterization of decreased bone mass, microstructure variation in bone tissue, and increased fracture risk [2]. As one of the cutting-edge research problems in the world, many efforts have been conducted to explore the pathogenesis of osteoporosis, as well as the development of treatment ([3]; Dai & Wang). Osteoporosis is a natural phenomenon of aging, whose incidence is related to various factors, such as age, hormone, nutrition, cytokines, and aging [4]. Bone tissue is constantly updated via the process of bone reconstruction participated by osteoblasts and osteoclasts, which mainly consists of four stages: activation, absorption, reversal, and bone formation. The pathological basis for osteoporosis is a negative mass balance of absorbed bone to new formatted bone during the procedure of bone reconstruction [5, 6].

MicroRNAs (miRNAs) are small, noncoding RNAs with 18 to 22 nucleotides that participate in posttranscriptional regulation of target gene expression by interacting with the mRNA 3′ nontranslational region (3′-UTR) of target gene, leading to mRNA degradation or translational inhibition ([7]; Thomas et al.). Numerous studies have shown that miRNAs are involved in the osteogenic differentiation process of BMSCs. For example, miR-26a is dependent on the unique activation and action of Wnt and bone morphogenetic protein (BMP) signaling pathways, which in turn enhances osteogenic differentiation of BMSCs [8]. By contrast, miR-30e represses osteogenic differentiation of BMSCs by targeting and downregulating insulin-like growth factor II [9]. Similarly, miR-124 inhibits expression of distal-less homeobox 5 (Dlx5), Dlx3, and Dlx2 to inhibit the osteogenic differentiation of BMSCs [10].

Many reports have indicated roles of miRNA-346-5p. Tsai et al. found that abnormal expression of miR-346-5p during pregnancy is closely related to various complications of pregnancy and fetus during pregnancy [11]. Peng et al. indicated that miR-346-5p regulates Wnt/*β*-catenin signaling to reduce the expression of downstream genes including c-Myc, CyclinD1, LEF-1, and TCF-1 and subsequent osteogenic differentiation of BMSCs [12]. Miao et al. found that miR-346-5p regulates the differentiation and proliferation of neuronal stem cells by regulating KLF4 expression [13]. However, the function of miR-346-5p in osteogenic differentiation of BMSCs is still not clear.

As a novel glycoprotein, TMEM9 contributes to liver regeneration and tumorigenesis [14, 15]. However, whether TMEM9 is involved in osteoblast differentiation of BMSCs remains unknown. Thus, the primary aim of this study was to investigate the effect of miR-346-5p and TMEM9 in osteogenic differentiation of BMSCs and to elucidate whether TMEM9 was a target of miR-346-5p.

## 2. Materials and Methods

### 2.1. Cell Culture

Human BMSCs purchased from Invitrogen (Carlsbad, CA, USA) were inoculated onto T75 flask and cultured with Dulbecco's modified Eagle medium (DMEM) containing 10% fetal bovine serum (FBS) and 1% penicillin/streptomycin (all from Hyclone, Logan City, Utah, USA). The cells were cultured at 37°C in a humidified atmosphere with 5% CO_2_.

### 2.2. Cell Transfection

The miR-346-5p inhibitor, miR-346-5p mimics, and the corresponding negative control (NC) were obtained from GenePharma (Shanghai, China). In addition, Lipofectamine 2000 (Invitrogen, Eugene, Oregon, USA) was used for transfections of miR-346-5p inhibitor (50 nM), miR-346-5p mimics (50 nM), and corresponding negative controls according to the manufacturer's requirement.

### 2.3. Osteogenic Differentiation and Staining In Vitro

Human BMSCs with 70-80% confluency were replaced conventional growth medium to osteogenic differentiation medium (high-glucose DMEM supplemented with 10% FBS, 1 nM phlegm, 10 mM *β*-glycerophosphate, and 0.2 mM l-ascorbic acid). Osteogenic differentiation medium was replaced every 3 days for 15 days. Next, the osteoblast phenotype was assessed by ALP staining using the ALP staining kit (Chinese Academy of Medical Sciences, Shanghai, China) according to the manufacturer's requirement. Moreover, 2% ARS provided by Sigma-Aldrich (Darmstadt, Germany) was utilized to identify matrix mineralization followed by an Olympus IX73 inverted microscope (Olympus, Tokyo, Japan).

### 2.4. qRT-PCR

Total RNAs from BMSCs were extracted by TRIZOL reagent (Invitrogen). Subsequently, cDNA was synthesized by reverse transcription utilizing the High-capacity RNA-to-cDNA Kit (ABI, Forest City, CA, USA). The SYBR qRT-PCR kit (TaKaRa, Dalian, China) was used for the detection of mRNA expression. Moreover, reaction conditions used for qRT-PCR were as follows: predenaturation at 95°C for 15 min, total 40 cycles of deformation at 95°C for 5 s, and annealing at 60°C for 15 sec. GAPDH was used as the endogenous control for mRNA. The relative expression amount of mRNA = 2^−ΔΔCt^∗100%.

### 2.5. Western Blot Analysis

Levels of targeted proteins were examined by Western Blot using monoclonal antibodies against Osterix, Runx2, and TMEM9 proteins (1 : 1000, Nanjing Kaiji Biological Development Co., Ltd., Nanjing, China). GAPDH (1 : 5000, Nanjing Kaiji Biological Development Co., Ltd.) was served as a loading control. After the incubation with primary antibodies, a horseradish peroxidase-labeled secondary antibody (1 : 3000, Nanjing Kaiji Biological Development Co., Ltd.) was used and incubated with the PVDF membrane (Millipore, Burlington, MA, USA) for 1 h at room temperature. Quantification of band density was performed using ImageJ (NIH Image, Bethesda, MD, USA).

### 2.6. Luciferase Reporter Assay

The wild-type (WT) TMEM9 mRNA 3′-UTR with miR-346-5p putative binding site and mutant (MUT) TMEM9 mRNA 3′-UTR without miR-346-5p putative binding site were cloned into the pmirGLO reporter vectors. Next, the reporter vectors containing WT or MUT 3′-UTR of TMEM9 mRNA were cotransfected with miR-346-5p mimic or mimic NC into HEK293T cells. After 48 hours of transfection, the activities of luciferase normalized to Renilla luciferase was detected by the Dual-Luciferase Assay System (Promega, Madison, WI, USA).

### 2.7. Statistical Analyses

GraphPad 8.0 software was used for the statistical analysis. All experiments were repeated triple times, and the data were presented as mean ± standarddeviation (SD). Statistical analyses were carried out using analysis of variance (ANOVA). *P* < 0.05 of data was considered significantly.

## 3. Results

### 3.1. MiR-346-5p Suppresses Osteogenic Differentiation of BMSCs

Results of the ALP and ARS staining indicated that miR-346-5p overexpression significantly decreased ALP activity and calcium deposition compared to those in cells transfected with mimic NC at day 7 and day 14 after being differentiated (indicated by white arrows; Figures 1(a) and 1(b)). By contrast, silence of miR-346-5p by inhibitors dramatically increases ALP activity and calcium deposition in BMCSs at day 7 and day 14 after being differentiated (indicated by white arrows; Figures 1(a) and 1(b)). The above results suggested that miR-346-5p suppressed osteogenic differentiation of BMSCs.

### 3.2. miR-346-5p Regulates the Expression of Key Osteoblast Markers during Osteoblast Differentiation

Next, we questioned whether miR-346-5p blocks the expression of transcription factors (Osterix and Runx2) involved in osteoblast differentiation. Results indicated that miR-346-5p overexpression reduced the expression of the osteoblastic markers Osterix and Runx2 compared to those in cells treated with mimic NC at day 7 and day 14 after being differentiated (Figures 2(a) and 2(b)). Instead, silence of miR-346-5p by an inhibitor promoted the expression of Osterix and Runx2 compared to those in cells treated with inhibitor NC at day 7 and day 14 after being cultured with osteogenic differentiation medium (Figures 2(a) and 2(b)). These results further suggested that miR-346-5p suppressed osteogenic differentiation of BMSCs.

### 3.3. miR-346-5p Directly Targets TMEM9

According to TargetScan analyses, there is a putative binding site of miR-346-5p mapped to TMEM9 mRNA 3′-UTR, suggesting that TMEM9 is a candidate target gene of miR-346-5p (Figure 3(a)). To further identify whether miR-346-5p directly targets TMEM9, luciferase reporters containing either the WT TMEM9 mRNA 3′-UTR or the MUT TMEM9 mRNA 3′-UTR were used (Figure 3(a)). Results showed that overexpression of miR-346-5p reduced luciferase activity of TMEM9 compared with that in cells treated with mimic NC (Figure 3(a)). In addition, miR-346-5p mimics did not affect the luciferase activity of TMEM9 containing the mutated miR-346-5p binding site (Figure 3(a)). Furthermore, data of Western Blot showed that overexpression of miR-346-5p dramatically decreased the protein level of TMEM9 compared to that in cells transfected with mimic NC, whereas silence of miR-346-5p by inhibitor increased the level of TMEM9 protein (Figure 3(b)). These data suggested that miR-346-5p directly targeted TMEM9.

## 4. Discussion

The current study indicated that miR-346-5p played a negative role in the osteogenic differentiation of BMSCs. Moreover, results of this study suggested that miR-346-5p in BMSCs inhibited osteogenic differentiation through targeting TMEM9.

miRNAs are a small class of noncoding RNAs which regulate expression of target genes at a posttranscriptional level. Previous studies have revealed that microRNAs play a crucial role in the differentiation of BMSCs into osteoblasts. For example, during osteoblast differentiation of BMSCs, miR-138 is reduced to activate the focal adhesion kinase- (FAK-) extracellular signal-regulated kinase 1/2 (ERK1/2) signaling pathway [16]. Moreover, miR-20a enhances osteogenic levels of BMSCs through activating BMP-Runx2 pathway by downregulating peroxisome proliferator-activated receptor-gamma (PPAR*γ*), BMP, and activated membrane-bound inhibitor homologs (Bambi) and cysteine-rich motor neurons 1 protein (Crim1) [17]. In addition, the ALP in osteoblast helps to produce phosphoric acid, which could react with Ca^2+^ to generate calcium phosphate deposits. Therefore, the ALP activity is an important factor for the osteoblast cells [18]. For miR-346-5p, our results revealed that upregulated miR-346-5p markedly decreased ALP activity and calcium deposition at day 7 and day 14 after being differentiated. However, a significant increase of ALP activity and calcium deposition was observed in BMSCs transfected with miR-346-5p inhibitors at day 7 and day 14 after being differentiated.

Osterix and Runx2 are important proteins involved in the proliferation process of osteoblasts. Osterix is essential for bone formation both in young ones and in adults [19] by regulating the expression of genes involved in the homeostasis of cortical bone [20]. As a transcription factor, Runx2 enhances osteoblastic proliferation and skeletal morphogenesis and serves as a scaffold for noncoding RNAs and regulatory factors contributed to skeletal gene expression (Shui et al.; [21]). Results of our study revealed that protein levels of the osteoblastic markers Osterix and Runx2 were decreased in BMSCs treated with miR-346-5p mimics at day 7 and day 14 after being differentiated. By contrast, silence of miR-346-5p by an inhibitor increased protein levels of Osterix and Runx2. Thus, these data suggested that miR-346-5p suppressed osteogenic differentiation of BMSCs.

TMEM9 is an important glycoprotein, which localizes to the lysosomal membrane and is partially present on the early endosome membrane [22]. Recent studies have indicated that TMEM9 contributes to liver regeneration and tumorigenesis through regulating Wnt/*β*-catenin signaling [14, 15]. Besides, TMEM9 is essential for the production of proinflammatory factors and is involved in the tumor necrosis factor (TNF) signaling pathway (Dodeller *et al.*). Though the role of TMEM9 in osteogenic differentiation is unknown, previous studies have revealed the effect of glycoprotein on osteogenic differentiation. For instance, glycoprotein neural epidermal growth factor-like (NEL) protein 1 (NELL-1) induces osteogenic differentiation of MSC through activating Runx2 by promoting its phosphorylation, which in turn upregulates NELL-1 expression [23, 24]. Furthermore, laminin suppresses the early stage of osteogenic differentiation by integrin-*α*2/-*β*1 whereas it induces late osteogenic differentiation via the FAK/ERK pathway in dental follicle cell [25]. Therefore, TMEM9 may contribute to osteogenic differentiation.

Through the bioinformatics analysis of TMEM9 gene by TargetScan website, we found that there is a putative binding site of miR-346-5p mapped to TMEM9 mRNA 3′-UTR. Moreover, a dual luciferase reporter assay demonstrated that TMEM9 was a direct target of miR-346-5p. In addition, data of Western Blot showed that the protein level of TMEM9 was significantly reduced by miR-346-5p mimics. The results also indicated that silence of miR-346-5p by an inhibitor improved the protein levels of TMEM9. These results suggested that miR-346-5p may inhibit osteogenic differentiation of BMSCs through targeting TMEM9. However, further studies focused on the mechanism how TMEM9 regulates osteogenic differentiation were required.

Previous studies have indicated that TMEM9 regulates Wnt/*β*-catenin signaling pathway [14, 15]. In fact, Wnt/*β*-catenin signaling plays an important role in osteogenic differentiation. A recent study has revealed that TIMP-1 suppresses osteogenic differentiation of human BSMCs through inactivating Wnt/*β*-catenin signaling and subsequent Runx2 expression [26]. By contrast, adiponectin promotes BMSC osteogenic differentiation through activating Wnt/*β*-catenin signaling [27]. These studies suggest that TMEM9 may facilitate BMSC osteogenic differentiation by regulating Wnt/*β*-catenin signaling.

In summary, miR-346-5psuppressed osteogenic differentiation of BMSCs by targeting TMEM9, which may provide novel targets for the treatment of bone injuries.

## Figures and Tables

**Figure 1:** miR-346-5p inhibited osteogenic differentiation of BMSCs. (a) ALP activities of BMSCs in different samples and seeded on TCP for days 7 and 14 after being differentiated (magnification, ×100). (b) ARS staining for days 7 and 14 after being differentiated (magnification, ×100) and quantitative analyses of the mineralization of BMSCs of ARS staining. *N* = 3. ^∗^*P* < 0.05 vs. the mimic NC group; #*P* < 0.05 and ##*P* < 0.01 vs. the inhibitor NC group.

**Figure 2:** miR-346-5p suppressed expression of Osterix and Runx2. The expression of Osterix and Runx2 was determined by Western Blot at day 7 (a) and day 14 (b) after being differentiated. *N* = 3. ∗*P* < 0.05 and ∗∗*P* < 0.01 vs. the mimic NC group; #*P* < 0.05 and ##*P* < 0.01 vs. the inhibitor NC group.

**Figure 3:** miR-346-5p directly targeted TMEM9 and inhibited the expression of TMEM9. (a) Putative miR-346-5p binding sequence in the TMEM9 mRNA 3′-UTR and the mutated sequence of TMEM9 mRNA 3′-UTR. (b) Protein levels of TMEM9 were assessed by Western Blotting. *N* = 3. ^∗∗∗^*P* < 0.001 vs. the mimic NC group; ^##^*P* < 0.01 vs. the inhibitor NC group.

## Data Availability

All data, models, and code generated or used during the study appear in the submitted article.

## Abbreviations

ALP: Alkaline phosphatase
Bambi: BMP and activated membrane-bound inhibitor homologs
BMP: Bone morphogenetic protein
BMSC: Bone marrow-derived mesenchymal stem cell
Crim1: Cysteine-rich motor neurons 1 protein
DMEM: Dulbecco's modified Eagle medium
FAK: Focal adhesion kinase
FBS: Fetal bovine serum
IL-1: Interleukin-1
miRNA: MicroRNA
MUT: Mutant
NC: Negative control
NELL-1: Neural epidermal growth factor-like (NEL) protein 1
PPAR*γ*: Peroxisome proliferator-activated receptor-gamma
Runx2: Runt-related transcription factor 2
TMEM9: Transmembrane Protein 9
SD: Standard deviation
TLR: Toll-like receptors
TNF: Tumor necrosis factor
WT: Wild-type
3′-UTR: 3′ nontranslational region
